The article "Design of Integrated Management System of IPE Instructional Resources Information Based on Artificial Intelligence Environment" was retracted in 2023. Reasons: unreliable results or conclusions; concerns about the data; concerns about the results or conclusions; concerns about the peer review.

# Design of Integrated Management System of IPE Instructional Resources Information Based on Artificial Intelligence Environment

**DOI:** 10.1155/2022/4594090

**Published:** 2022-08-31

**Authors:** Duo Wang

**Affiliations:** School of Marxism, Xi'an University, Xi'an 710065, China

## Abstract

With the development of modern networks and their fast and convenient characteristics, the construction of instructional resources has become the focus of information construction in universities. Based on AI (Artificial intelligence) technology, this paper discusses the software development technology used in the comprehensive management system of IPE instructional resources. According to the application environment and application objects of the system, a comprehensive information management system of IPE instructional resources based on AI technology is constructed. In this paper, a concept similarity algorithm based on semantic similarity and semantic correlation is proposed to calculate the distance between words and establish concept mapping pairs. The semantic analysis of the information input by students is realized, and the proposed concept similarity algorithm is used in the domain ontology knowledge base to search for similar courses and recommend them to students for their choice. The test results show that the stability of this system can reach about 96%, which is about 10% higher than other systems. The comprehensive management system of instructional resources information proposed in this paper will promote educators and learners to find high-quality IPE instructional resources.

## 1. Introduction

The advent of AI has altered how people think and interact with one another, as well as given rise to new technical tools and strategies for social advancement. As a result of AI, learning methods are changing continuously along with the development of teaching materials [1]. The transition from single paper textbooks to “textbooks + digital resources” new media textbooks is a process that is also increasing the degree of informationalization of teaching and learning techniques. As there are more and more different kinds of network-based educational resources, network-based resource management is becoming more and more important and well-liked [2]. The creation of top-notch courses in universities will unquestionably be encouraged by instructional resources. IPECU (Ideological and Political Education in Colleges and Universities) primarily refers to the social practice activities of influencing and educating college students' attitudes, actions, and political viewpoints while working within the confines of pertinent rules and regulations established by colleges and education departments [3]. Planning and organization go into this type of practice. Its development urgently requires the effective support of network instructional resources because it is a component of IPE theory courses taught in universities. However, the way that educational resources are currently managed and used in universities is not optimal. Universities work to establish the appropriate instructional resources management system by utilizing computer and network technology in order to make the best use of the instructional resources in universities and to be used by teachers and students. Building an educational resource management system that satisfies the needs of teaching is essential because network resource management has taken on a completely new form. However, the majority of resource libraries are still isolated and dispersed, making it challenging to share and reuse due to the absence of uniform resource description standards and construction standards. A number of new changes have been made to the research paradigm, method, carrier, and environment of the subject and object of IPECU against the backdrop of AI [4, 5]. Therefore, discussing the comprehensive information management system of IPE instructional resources based on AI technology has some theoretical and practical significance.

The article "Design of Integrated Management System of IPE Instructional Resources Information Based on Artificial Intelligence Environment" was retracted in 2023. Reasons: unreliable results or conclusions; concerns about the data; concerns about the results or conclusions; concerns about the peer review.

The challenges that traditional IPE education faces can be effectively resolved by the advancement of information technology. IPE education can be better promoted, and the issues with the current IPE education resources in universities can be resolved through the development of a comprehensive information management system for IPE education resources [6]. In order to fully utilize network resources in IPE classroom teaching in universities and take advantage of the dominance of the development of the network era, IPE teachers who are at the forefront of IPE education for college students must also be clear about the definition and characteristics of IPE teaching network resources [7]. AI presents IPECU with both opportunities and challenges, but it also introduces some brand-new issues. Education that incorporates AI can actually achieve “teaching students in accordance with their aptitude” and raise the standard of IPECU [8]. This paper develops new ideas regarding the method of precise IPECU penetration and the tactic of integrating educational resources on the basis of the background of AI. The comprehensive management system of IPE instructional resources uses software development technology as its foundation, and this paper also discusses AI technology as a starting point. A comprehensive information management system of IPE instructional resources based on AI technology is built in accordance with the application environment and application objects of the system.

The article "Design of Integrated Management System of IPE Instructional Resources Information Based on Artificial Intelligence Environment" was retracted in 2023. Reasons: unreliable results or conclusions; concerns about the data; concerns about the results or conclusions; concerns about the peer review.

This paper mainly studies the design and application of a comprehensive information management system of IPE instructional resources based on AI. Its innovations are as follows:

① Based on AI technology, this paper discusses the software development technology used in the comprehensive management system of IPE instructional resources and puts forward the development scheme of the comprehensive management system of IPE instructional resources according to the system application environment and application objects.
② In this paper, a concept similarity algorithm based on semantic similarity and semantic correlation is proposed to calculate the distance between words and establish concept mapping pairs. The semantic analysis of the information input by students is realized, and the proposed concept similarity algorithm is used in the domain ontology knowledge base to search for similar courses and recommend them to students for their choice. At the same time, the system integrates instructional resources and innovates teaching methods. After testing, it runs stably, operates simply, and has a clear interface, which can meet the teaching needs of universities.

## 2. Related Work

The Internet has provided conditions for the innovation and development of IPECU, and the organic combination of the two has radiated infinite vigor and vitality. Scholars have conducted extensive discussions on the laws, contradictions, mechanisms, and methods of IPE education. They have paid equal attention to theoretical exploration and practical application. They have accumulated certain achievements and formed a relatively mature theoretical framework and research paradigm. Deng and Wang analyzed the current situation of IPE instructional resources in universities and designed a practical teaching network platform based on the integration of IPE instructional resources in universities [9]. Guided by constructivist learning theory and network communication theory, Lu [10] discussed strengthening the teaching of IPE courses in universities from the basic principles, technology expansion, platform construction, team building, and other aspects of the construction of network instructional resources for IPE courses in universities. The effective way of resource construction put forward corresponding countermeasures [10]. Li believes that, based on the current situation, online teaching is only suitable for some specific teaching content and for students with strong self-control ability, so online teaching can only be used as an effective supplement to classroom teaching but cannot be used as a substitute for classroom teaching [11]. Tian [12] combines the SQL Server database management system to design and develop the instructional resource management system. Its purpose is to implement efficient and unified management of educational resources so that teachers and students can make full use of them [12]. Dong and Chen believe that the characteristics of traditional classroom teaching are that the knowledge of textbooks, teachers, and lesson plans are the basis, which fundamentally lacks the overall care for students [13]. Zhang [14] discusses the research and implementation of an instructional resource management system based on learning object metadata. Through specific analysis, research, and implementation, it provides system support for the construction of a standardized resource library [14]. On the premise of introducing the concepts of Semantic Web and Ontology and their key technologies, Lin, with the help of domain experts, constructed an ontology knowledge base in the field of instructional resource management according to the rules of ontology construction [15]. Kardan et al. [16] conducted an in-depth analysis and research on the instructional resource management system in universities. It mainly discusses user requirements, functional requirements, feasibility analysis, and hardware configuration and finally determines that the functional module of the system consists of four parts: user management, resource service, resource management, and system management [16]. Su et al. pointed out that there is a discourse dilemma in the classroom teaching of IPE courses in universities; the discourses of IPE course teachers are relatively old, not vivid enough, the theory is divorced from reality, and it lacks persuasiveness and appeal [17].

The article "Design of Integrated Management System of IPE Instructional Resources Information Based on Artificial Intelligence Environment" was retracted in 2023. Reasons: unreliable results or conclusions; concerns about the data; concerns about the results or conclusions; concerns about the peer review.

For IPECU, AI is both an opportunity and a challenge, but it also brings some new problems. In the past, network instructional resources were insufficient and the quality was not high. There were an emphasis on content construction, neglect of application effect, and insufficient interaction between teachers and students. Based on this, this paper takes AI technology as the starting point and discusses the software development technology adopted by the comprehensive management system of IPE instructional resources. According to the application environment and application objects of the system, a comprehensive information management system of IPE instructional resources based on AI technology is constructed. Among them, strengthening the overall planning and management of instructional resources in schools, making efforts to tap and utilize hidden educational resources, and giving full play to students' main roles are the main strategies to systematically integrate the instructional resources of IPE courses. The construction of the system makes IPE instructional resources effectively managed and utilized, better meets the needs of teachers and students, and serves education and teaching better.

## 3. Methodology

### 3.1. Strategies for Integrating Instructional Resources in the AI Environment

Under the background of AI, the educational goal will put more emphasis on the cultivation of higher-order thinking. People's values and information literacy are likely to have some changes under the influence of intelligent technology, which will present a new teaching form. With the continuous improvement of information technology [18, 19] level, the integration of network and people's life has improved, and college students' interest and attention to the network has increased significantly. Although different organizations and departments have established departmental websites, they all have the problems of a single form and monotonous content. This will reduce students' interest in these websites, resulting in a relatively low utilization rate of teaching information resources of IPECU. Only by integrating all kinds of instructional resources in a diversified way and then rationally allocating and efficiently using them can we complete teaching activities and achieve the overall goal of educating people, thus expanding the scope and improving the level of IPE teaching. IPE educators in universities can make use of the advantages of AI technology in situation creation and man-machine interaction and help students to change their knowledge from the superficial theoretical study of IPE education to practical application of IPE education. To strengthen and innovate the teaching of IPE courses, we must first master sufficient instructional resources. The IPE theory course covers a wide range of contents and has the characteristics of profound theory, prominent politics, and key practicality. The sharing of online instructional resources can meet the needs of teachers and students for diverse, timely, and efficient teaching and learning resources. Compared with off-campus resources, the utilization of on-campus resources is more independent, convenient, and feasible, the cost of development and integration is lower, and there is more room for innovation. The integration and utilization of available resources in schools can greatly alleviate the practical difficulties of the lack of IPE instructional resources. We should ensure the sharing of excellent instructional resources in universities, but we should develop the resources at a later period. When developing instructional resources, we must ensure that there is a sound incentive mechanism for students' growth. At the same time, teachers of IPE courses in universities need to grasp the principles and norms of network resources utilization, follow the principle of political orientation, and always reflect the correct political direction; follow the principle of innovation and always adhere to the spirit of innovation; follow the scientific principle and give consideration to the attractiveness and systematicness of classroom teaching; and follow the principle of comprehensiveness, correctly use positive and negative network resources, and constantly improve the standardization and rationality of network resource utilization. The biggest feature of AI is intelligence. The integration of AI and education has changed the situation of large-scale training of mechanized and standardized talents in the past, and the teaching methods are gradually becoming intelligent. AI has made great progress, can adapt to a variety of personalized needs, and has the ability of self-study. In the teaching methods of IPECU, AI will become the key force that affects its development.

The article "Design of Integrated Management System of IPE Instructional Resources Information Based on Artificial Intelligence Environment" was retracted in 2023. Reasons: unreliable results or conclusions; concerns about the data; concerns about the results or conclusions; concerns about the peer review.

The construction of network instructional resources for IPE theory courses in universities is conducive to sharing network instructional resources, innovating network teaching methods, and improving the effectiveness of network teaching of IPE theory courses in universities. Focusing on the teaching objectives of IPE courses, scientifically organizing, rationally developing, coordinating, and optimizing the existing or potential instructional resources of IPE courses in universities in accordance with the laws and objective conditions of education and teaching is what it means to integrate the instructional resources of IPE courses in schools. This allows all the human, material, and financial resources of universities with IPE education value to serve the teaching. When conducting IPE education courses, the school's resources play a crucial role [20]. Universities can adhere strictly to the principles of one team, overall management, clear paths and rivers, and scientific use and can distribute IPE educators in a rational and scientific manner. The effective realization of the sharing of IPE instructional resources in universities is strengthened by the integration of teaching human resources, which also improves communication and cooperation among various organizational departments in universities. These functional modules have also increased the level of interaction between teachers and students. Examples include interactive platforms, student work display platforms, entrepreneurship and employment, and practical teaching quality effect evaluation. The use of the teaching network platform by students in this interactive setting increases their willingness to do so, which raises the rate at which actual teaching information resources are used. The key to applying big data and AI technology in higher education is to gather data on how students learn, as this is a crucial way to support personalized learning for all students. It is clear that any effort to promote the study of scientific methodology in the educational system will undoubtedly be fruitful. The emergence of intelligent tutoring systems and AI-adaptive education systems has upset the balance of knowledge dissemination in IPE education and encouraged students to cultivate the habit of autonomous learning, which makes them more engaged in their studies. We should revise the educational model in light of this, and we should modify how we use network resources. In order to realize the rational utilization of network resources and effectively improve the allure, appeal, pertinence, and effectiveness of classroom teaching of IPE courses in universities, the network position should be strengthened and the environment of IPE resources usage should be optimized as a path to promotion. In the process of establishing a diversified instructional resource system, we should do the following: ① strengthen the integration of IPE practice instructional resources and ② establish a teacher linkage system, that is, to strengthen the connection between teachers and ensure that the IPE course education can be adjusted in time according to the current social development and the actual needs of school development. Through integration, all kinds of tangible and intangible resource elements will form an organic, harmonious, and unified resource system, which will help to form the joint force of IPE education and ensure the integrity and long-term effectiveness of IPE education.

The article "Design of Integrated Management System of IPE Instructional Resources Information Based on Artificial Intelligence Environment" was retracted in 2023. Reasons: unreliable results or conclusions; concerns about the data; concerns about the results or conclusions; concerns about the peer review.

### 3.2. Design of the Comprehensive Information Management System for IPE Instructional Resources

IPE educators in universities must analyze the current changes from a big data perspective, digitize the IPE education work, and use big data thinking to make more sensible decisions in light of AI. The development of an extensive information management system for IPE instructional resources can achieve the efficient linking of learning resources, including information resources and wisdom resources, and the formation of a wisdom community. It can also achieve the creation of an open learning community and realize the material guarantee of ecological learning. It is inevitable that students will run into some sort of difficulty while studying IPE theory. Through online communication and in-person consultation on the platform of instructional resources, teachers' theoretical guidance can be obtained, helping to close the gap between them and their students while also encouraging their study of IPE theory. The discussion and exchange between students also reflect college students' experiences, which facilitates a quicker and more convenient exchange of ideas. The system supports teaching and learning, improves the effectiveness of the use of instructional resources, completes their effective management, enables teachers and students to use a variety of resources for quick searches and reading, assists them in continuing their studies after school, and fosters their growth as independent learners. Deepening and fine-tuning the system requirements analysis is the process of system design. In order to ensure the security, dependability, and high efficiency of the system, it is essential to adopt a rational and scientific system design approach from the system's implementation environment. Relevant staff should concentrate on combining the actual situation of universities and excavating and integrating various IPE instructional resources in universities when designing the comprehensive information management system of IPE instructional resources. The system structure and modules are shown in Figure 1.

The system design of this paper mainly follows the following principles. ① *Clarity*. The system should be concise, clear, and comfortable. ② *Practicality*. The functional design of the system should be complete and well realized, which can meet the operating needs of teachers and students. ③ *Simplicity*. In the process of system design, the convenience and feasibility of system operation should be fully considered. ④ *Interaction*. The system should have a good interactive function, which is convenient for teachers and students to explore, so as to continuously enhance their cooperative learning ability. ⑤ *Common Normative Principle*. Instructional resource management system follows unified norms and principles. The overall design is mainly divided into functional modules of the system. After fully analyzing the internal requirements of the system, it is concluded that the system consists of six functional modules: user management module, resource editing module, resource management module, resource retrieval module, resource evaluation module, and element set introduction module.

There are three steps in the resource recommendation process: one is to establish an evaluation matrix; the second is to find the nearest neighbor of the target resource by the similarity; the third is to form a recommendation. The evaluation matrix is as follows:

(1) $$\begin{array}{c} A\left(m,n\right)=\left[\begin{array}{ccccc} A_{1,1} & A_{1,2} & A_{1,3} & \cdots & A_{1,n}\\ A_{2,1} & A_{2,2} & A_{2,3} & A_{2,n}\\ \cdots & \cdots & \cdots & \cdots & \cdots \\ A_{m,1} & A_{m,2} & A_{m,3} & \cdots & A_{m,n} \end{array}\right]. \end{array}$$

Cosine similarity: in the matrix, resources can be regarded as *m*-dimensional vectors, and the cosine angle between vectors can be used to find the similarity between resources. A larger value means a higher degree of approximation between resources. The formula is as follows:

(2) $$\begin{array}{c} \text{Sim}\left(i,j\right)=\cos\left(\bar{i},\bar{j}\right)=\frac{\bar{i}\cdot \bar{j}}{\left\|\bar{i}\right\|\cdot \left\|\bar{j}\right\|}. \end{array}$$

Pearson product-moment correlation coefficient: find the correlation degree of two vectors and find the similarity between them. The greater the absolute value of this coefficient, the stronger the correlation. The formula is as follows:

(3) $$\begin{array}{c} \text{Sim}\left(i,j\right)=\frac{\sum_{a\in U}\left(A_{a,i}-{\bar{A}}_{i}\right)\left(A_{a,j}-{\bar{A}}_{j}\right)}{\sqrt{\sum_{a\in U}{\left(A_{a,i}-{\bar{A}}_{i}\right)}^{2}}\times \sqrt{\sum_{a\in U}{\left(A_{a,j}-{\bar{A}}_{j}\right)}^{2}}}. \end{array}$$

In the formula, *A*_*a*,*j*_ is the score of the resource *j* given by the user *a*; ${\bar{A}}_{i}$ is the average of the *i* th resource scored by the user *a*; ${\bar{A}}_{j}$ is the average of the *j* th resource scored by the user *a*. Recommendations are formed by judging *P*_*a*,*i*_ on the target knowledge content. The relevant formula is

(4) $$\begin{array}{c} P_{a,i}=\frac{\sum_{\text{similar}-\text{items},k}\left(T_{i,k}*A_{a,k}\right)}{\sum_{\text{similar}-\text{items},k}\left(\left|T_{i,k}\right|\right)}. \end{array}$$

In the formula, *A*_*a*,*k*_ is the score of the similar resource *k* by the user *a*; *T*_*i*,*k*_ is the approximation of the target resource *i* and the nearest neighbor *k*.

The article "Design of Integrated Management System of IPE Instructional Resources Information Based on Artificial Intelligence Environment" was retracted in 2023. Reasons: unreliable results or conclusions; concerns about the data; concerns about the results or conclusions; concerns about the peer review.

Assuming two concepts Con1 and Con2 in the ontology, the degree of similarity between these two terms is Sim(Con1, Con2). Then, there is the following formula:

(5) $$\begin{array}{c} \text{Sim}\left(\text{Con}1,\text{Con}2\right)=\sum_{i=1}^{n}\theta_{i}\left(\text{Con}1,\text{Con}2\right)\sigma_{i}. \end{array}$$

Among them, *n* is the maximum depth of the term in the ontology concept model; *σ*_*i*_ represents the weight. The value of *θ*_*i*_(Con1, Con2) is defined as follows: when the first *i* parent classes of Con1 and Con2 are the same:

(6) $$\begin{array}{c} \theta_{i}\left(\text{Con}1,\text{Con}2\right)=1. \end{array}$$

When the first *i* parent classes of Con1 and Con2 are different:

(7) $$\begin{array}{c} \theta_{i}\left(\text{Con}1,\text{Con}2\right)=0. \end{array}$$

The way to calculate the concept of semantic distance is as follows: Dis(Con1, Con2)=Con1‘s superclass list length + Con2‘s superclass list length. The semantic similarity is calculated as follows.

Assuming that there are two concepts Con1 and Con2 in the ontology, and the degree of similarity between these two terms is SSim(Con1, Con2), there is the following formula:

(8) $$\begin{array}{c} \text{SSim}\left(\text{Con}1,\text{Con}2\right)=\frac{\sum_{i=1}^{n}\theta_{i}\left(\text{Con}1,\text{Con}2\right)}{\text{Dis}\left(\text{Con}1,\text{Con}2\right)}\\ +\min\left(\frac{\sum_{j=1}^{m}\phi_{i}\left(\text{Con}1,\text{Con}2\right)}{\max\left(\text{Len}C\left(\text{Con}1\right),\text{Len}C\left(\text{Con}2\right)\right)},0.5\right). \end{array}$$

Among them, AA is the maximum depth of concept BB and concept CC in the ontology concept model; DD is the maximum number of subclasses of concept BB and concept CC in the ontology concept model; EE represents the semantics between concept BB and concept CC Distance; FF represents the number of all subclasses of concept GG.

Among them, *n* is the maximum depth of concept Con1 and concept Con2 in the ontology concept model; *m* is themaximum number of subclasses of concept Con1 and concept Con2 in the ontology concept model; Dis(Con1, Con2) represents the semantics between concept Con1 and concept Con2 Distance; Len*C*(Con) represents the number of all subclasses of concept Con.

The design of digital instructional resources follows the general method of teaching system design, and at the same time, the characteristics of digital instructional resources should be taken into account: the sources are complex and diverse, and there are great differences among learners, so the design should be classified according to the specific situation. The system has two functions: one is the function of the front desk; the second is the function of the background. Among them, the foreground is completed by ASP.NET development tools, while the background is managed by SQL Server. In addition, this paper uses the *Eucalyptus* platform to obtain the interface in the form of Web service through public API to develop the application software of the network platform and create the service cloud of practice teaching and integrate virtualization technology, server clusters, and storage devices to support the processing and service application of massive instructional resources, so as to provide cloud service support for IPE practice teaching. The cloud service platform of California is shown in Figure 2.

The article "Design of Integrated Management System of IPE Instructional Resources Information Based on Artificial Intelligence Environment" was retracted in 2023. Reasons: unreliable results or conclusions; concerns about the data; concerns about the results or conclusions; concerns about the peer review.

In the aspect of system manipulation of databases and data, it is necessary to create reliable guarantees such as data integrity, so as to ensure that the system does not run abnormally and firmly. At the same time, the system program interface is concise and simple, and the operation is convenient; There is also a way of searching, which allows teachers and students to quickly find the relevant knowledge they need by searching. The system provides simultaneous access for a large number of users, which is universal enough to enable all universities to provide educational services, and has scalability and fault tolerance. In this way, IPE teachers will play the role of interlocutor on the basis of the role of guide. In order to improve the recall and precision of information query and retrieval, the semantic analysis of information submitted by users should be done first. After that, the user's query requirements are semantically analyzed and converted into ontology representation. Finally, the domain ontology knowledge base can be retrieved. The normal, safe, and efficient operation of the system is inseparable from the good performance of the system. The following are the performance requirements of this system. ① *Ease of Use*. In order to effectively enhance the efficiency of teachers and students in using the system, we should not only consider the good functional layout of the system but also consider the good use experience of teachers and students. ② *High Performance*. ③ *Scalability*. Since knowledge is constantly updated and changing, we should try our best to consider its expansibility in the early stage of research and development. In addition, this paper uses two performance evaluation indexes to evaluate the effectiveness of the algorithm. They are MSE (Mean squared error) and MAE (Mean absolute error), respectively. The definitions of these two indicators are as follows:

(9) $$\begin{array}{c} MSE=\frac{1}{n}{\sum_{k=1}^{n}\left(y_{k}-y_{k}^{\prime }\right)}^{2},\\ MAE=\frac{1}{n}\sum_{k=1}^{n}\left|y_{k}-y_{k}^{\prime }\right|. \end{array}$$

Among them, *y*_*k*_ is the actual value, and *y*_*k*_′ is the output value.

This system uses the combination of a file management system and a relational database to realize the storage and management of instructional resources. The file system is used to store different instructional resources and their descriptive metadata, that is, documents, and the database is used to store key information that can completely describe resources, that is, core metadata information. Data information is kept in the database, all the data are disposed of in the database, and the database plays the role of manipulating all the data. The database is the core content of the system, and the design of the database plays a key role in development. In the design of the file system, firstly, according to the specific classification of media materials, five folders of text materials, graphic materials, audio materials, video materials, and animation materials are created, respectively, and then the resources and the documents describing them are stored in the corresponding folders according to the types of registered resources. After the system obtains the information submitted by the query engine, the semantic analysis component transforms the user's conceptual hierarchy into the ontology conceptual hierarchy, which simply means formalizing the user's query information ontology. Then, the Jena reasoning engine is used to analyze and reason the semantic query information, so that the query information can be understood and the search results can meet the user's query requirements.

The article "Design of Integrated Management System of IPE Instructional Resources Information Based on Artificial Intelligence Environment" was retracted in 2023. Reasons: unreliable results or conclusions; concerns about the data; concerns about the results or conclusions; concerns about the peer review.

## 4. Result Analysis and Discussion

For an application system, a concise and friendly user interface can facilitate users to use the system better. The system lists the menu of the system's functional modules according to the hierarchy, and the functional descriptions of the corresponding modules appear in the right column of the main interface in turn. The design of the navigation bar plays a very important role in the whole system construction, and it will directly affect whether users can get to the place they want to go and then easily complete their operations. In addition, this system implements structured data storage, so that teachers and students can achieve effective retrieval and then complete efficient access. The composition of the IPE education resources management database table is shown in Table 1.

Announcing, information statistics, friendship links, searches, and a variety of resources recently uploaded are all included in the system's main interface. The tree structure display on the left side of the result display interface displays the categories of courses primarily; the table structure display on the right side of the interface displays the detailed information related to the course, such as course similarity, course ID, course teachers, and knowledge points of the course. The management system can quickly query and manage educational resources scientifically thanks to the integration of a file management system and a relational database that ensures the integrity of metadata information. The goal of technical feasibility analysis is to determine whether the necessary technology, including the quantity and expertise of system developers, hardware, software, and other application technologies, is readily available to achieve the objectives of the new system.  Table 2 shows the software and hardware requirements of the system server.

The article "Design of Integrated Management System of IPE Instructional Resources Information Based on Artificial Intelligence Environment" was retracted in 2023. Reasons: unreliable results or conclusions; concerns about the data; concerns about the results or conclusions; concerns about the peer review.

Running a program to look for errors is called testing. A test that is likely to uncover errors that have not yet been discovered is referred to as a good test case. A test that is effective finds errors that have not yet been discovered. The experimental MSE of the algorithm results is shown in Figure 3. The experimental outcomes of the MAE algorithm are displayed in Figure 4.

It is clear that this algorithm has low MSE and MAE. This paper implements the key technology of data query as well as the addition, modification, and deletion of data information in order to enhance the functionality of the instructional resource management system. Response time is referred to as “system response time,” which primarily refers to the amount of time required by the application system between the time the request is sent and the time the objective end receives the response. Consider it to be the primary example of software performance from the user's point of view. On the assumption that the configured test environment can meet the requirements of system user response time, this paper tests the maximum number of concurrent users carried by the system as well as the response time of key services under a given amount of data. The response time test results of the system are shown in Figure 5.

In order to explore the influence of iteration times on the model, the values of other parameters were fixed during the experiment, including the basic learning rate and the number of batch pictures.  Table 3 shows the change in model accuracy when different iterations are set. Eight groups of data with iteration times ranging from 3,000 to 10,000 were selected to observe the change in model accuracy.

This section combines the system's core functions, namely, resource service and resource management, designs test cases for the system, tests the system appropriately, ensures the validity of the test results, and precisely assesses the system's performance. The system's stability test results are displayed in Figure 6.

The “Number of concurrent users” in Figure 6 refers to the number of customers making requests to the server at the same time. This concept is generally used in conjunction with concurrent testing, which reflects the maximum number of concurrent accesses borne by the server. It can be seen that the system in this paper can maintain good stability even when there are many concurrent users.

The table structure used in this paper is simpler than the tree structure. With regard to the structure of the table, we should first define the table style and a class for obtaining course information and then provide table Viewer with the tagger and inner container in SWT. The function of the content container is to extract a required object from all the course collection classes, while the function of the tagger is to extract a field in the course object information of a corresponding cell from a course object. Finally, in the main program of the result display interface, the relevant information about the course is displayed in tabular form. Batch number of pictures refers to that in the process of training, at the beginning of each iteration, a part of training data is selected first, and this part of data is the number of pictures processed by the network model in one iteration.  Figure 7 shows the change of the accuracy of the algorithm when setting different numbers of batch images.

The article "Design of Integrated Management System of IPE Instructional Resources Information Based on Artificial Intelligence Environment" was retracted in 2023. Reasons: unreliable results or conclusions; concerns about the data; concerns about the results or conclusions; concerns about the peer review.

It can be seen that with the increasing number of batch images, the accuracy rate will be continuously improved within a certain number of images. However, when the number of batch images exceeds a threshold, the influence of the value of the batch images on the accuracy will decrease, and the accuracy of the model tends to be stable.

After testing in this chapter, we know that the stability of this system can reach about 96%, which is about 10% higher than other systems. At the same time, the integrated management system of instructional resources information has a simple interface and simple operation, functions in line with expectations, and can meet the needs of users. After testing, the performance of the system has been greatly improved, and the quality of the instructional resource information integrated management system software has been improved, making the system more competitive in the market. The comprehensive management system of instructional resources information proposed in this paper will promote educators and learners to find high-quality IPE instructional resources.

## 5. Conclusions

From the perspective of IPE class teaching, network resources are all information resources that can be used in IPE class teaching in universities through the Internet. It has a huge capacity and rapid update and is rich in content and high in sharing. The rational use of network resources by political teachers in classroom teaching can meet the needs of expanding classroom capacity, meeting the needs of contemporary college students, responding to the challenge of negative network information, and meeting the requirements of the development of the network era. In view of the present situation of IPE instructional resources utilization, this paper puts forward the strategy of instructional resources integration under the AI environment. Among them, strengthening the overall planning and management of instructional resources in schools, making efforts to tap and utilize hidden educational resources, and giving full play to students' main roles are the main strategies to systematically integrate the instructional resources of IPE courses. At the same time, according to the application environment and application objects of the system, this paper constructs a comprehensive information management system of IPE instructional resources based on AI technology. The test results show that the stability of this system can reach about 96%, which is about 10% higher than other systems. The development and utilization of the comprehensive information management system of IPE instructional resources can maximize the sharing and integration of IPE instructional resources. It not only innovates the teaching methods but also has very important practical significance. The comprehensive management system of instructional resources information proposed in this paper will promote educators and learners to find high-quality IPE instructional resources. Although some functions of the system need to be further improved, the research on the key technologies of AI-based comprehensive management system of IPE instructional resources has strong theoretical and practical significance. The next step will be to continuously improve and improve the functions of the system.

The article "Design of Integrated Management System of IPE Instructional Resources Information Based on Artificial Intelligence Environment" was retracted in 2023. Reasons: unreliable results or conclusions; concerns about the data; concerns about the results or conclusions; concerns about the peer review.

## Figures and Tables

**Figure 1:** Structure and module diagram of the system.

**Figure 2:** *Eucalyptus* cloud service platform.

**Figure 3:** Experimental results of MSE of the algorithm.

**Figure 4:** Experimental results of MAE algorithm.

**Figure 5:** Response time test results of the system.

**Figure 6:** Stability test results of the system.

**Figure 7:** Changes in the accuracy of the algorithm.

**Table 1:** Composition of the library table of IPE instructional resources management.

Serial number	Table name	Related description
1	b_gly	Store the login identity information of the system administrator
2	b_yhb	Store detailed registration information and management permission information of ordinary users
3	b_zylx	Store information such as category names of five small categories of media materials
4	b_wbsc	Store key metadata element information of text material resources
5	b_xsc	Store key metadata element information of graphics/image material resources
6	b_ypsc	Store key metadata element information of audio material resources
7	b_spsc	Store key metadata element information of video material resources
8	b_zypz	Store the personal evaluation information of the resources used by ordinary users

The article "Design of Integrated Management System of IPE Instructional Resources Information Based on Artificial Intelligence Environment" was retracted in 2023. Reasons: unreliable results or conclusions; concerns about the data; concerns about the results or conclusions; concerns about the peer review.

**Table 2:** Server-side software and hardware requirements.

Condition	Requirements
CPU	Intel i5 processor; frequency: 3.0 GHz
RAM	8 GB and above
Hard disc capacity	500 GB or more
Installation system	Microsoft Windows, SQL Server

Other software	Microsoft NET Framework SDK
	Microsoft Visual Studio
	IIS6.0

**Table 3:** Accuracy of the model with different iteration times.

Iterations	Accuracy
3000	35%–65%
4000	45%–70%
5000	60%–70%
6000	70%–85%
7000	80%–90%
8000	30%–50%
9000	28%–80%
10000	30%–90%

## Data Availability

The data used to support the findings of this study are available from the corresponding author upon request.
